# Relationship Between Acute Stress Responses and Quality of Life in Chinese Health Care Workers During the COVID-19 Outbreak

**DOI:** 10.3389/fpsyg.2021.599136

**Published:** 2021-03-16

**Authors:** Lan Zhang, Rongjian Ji, Yanbo Ji, Min Liu, Renxiu Wang, Cuiping Xu

**Affiliations:** ^1^Department of Nursing, Shandong Provincial Qianfoshan Hospital, Shandong University, Shandong, China; ^2^School of Nursing, Shandong First Medical University, Shandong, China; ^3^School of Nursing, Shandong University of Traditional Chinese Medicine, Shandong, China

**Keywords:** acute stress, coronavirus, health care workers, quality of life, China

## Abstract

This study aimed to determine the relationship between acute stress and quality of life and explore their influencing factors on health care workers. A descriptive cross-sectional study was conducted, and a sample of 525 health care workers was recruited from 15 hospitals through a convenient sampling method. Participants completed an online self-report questionnaire to assess their acute stress and quality of life. Descriptive and multiple linear regression statistics were used for this analysis. The results regarding acute stress responses varied significantly among the differences in marital status, physical activity, work status, perceived risk of contracting COVID-19, and the expected duration of the pandemic. Moreover, a younger age, lack of physical activity, being a front-line medical staff, and higher acute stress scores indicated a worse quality of life. Healthcare workers’ acute stress was negatively correlated with their quality of life. Therefore, the authorities should pay special attention to health care workers’ mental health and provide them with timely protection during the pandemic.

## Introduction

The coronavirus disease 2019 (COVID-19), an acute respiratory disease caused by β-coronavirus, has spread worldwide since it first appeared in Wuhan, China, in December 2019 (Paules et al., 2020). As of June 26, 2020, more than 9.2 million confirmed cases and 470,000 deaths have been reported worldwide, including 85,119 confirmed cases and 4,647 deaths in China (World Health Organization, 2020). The World Health Organization (WHO) officially declared the COVID-19 pandemic a public health emergency of international concern on January 30, 2020, marking the third pandemic of coronavirus in the 21st century (Mahase, 2020).

To control the COVID-19 pandemic swiftly, health care workers throughout China actively participated in medical treatment, disease prevention, and logistics support. However, due to the shortage of personal protective materials in the early stages, the persistence of the disease, and the highly contagious nature of the COVID-19 virus, health care workers were at risk of being infected with COVID-19 (Van Doremalen et al., 2020). Previous studies have showed a link between chronic work-related stress among healthcare workers and post-traumatic stress disorder (Laposa et al., 2003; Robertson and Perry, 2010). Meanwhile, long work hours and high-pressure environments increase the physical and psychological stress among medical staff, leading to anxiety, depression, and, at worst, suicide (Goyal et al., 2020).

Quality of life (QoL) refers to an individual’s self-perception of goals, expectations, standards, and concerns in the context of different cultures and value systems (Kuyken et al., 1995). Traumatic life events have various psychological and physiological consequences, affecting an individual’s well-being and QoL (Garfin et al., 2018). For example, adults who experienced an earthquake exhibit acute stress symptoms, psychological distress, and maladaptive behaviors (Dorahy et al., 2016). Correspondingly, some studies reported that Ebola survivors suffered from various physical and mental sequelae (James et al., 2019). Most existing studies have focused on the victims of COVID-19. Furthermore, several studies have explored the mental health and QoL of health care workers during the outbreak. In their systematic review, de Pablo et al. (2020) summarized that 62.5% of health care workers reported general health concerns during the outbreak of SARS, MERS-CoV, and COVID-19. Adverse psychological responses such as high levels of anxiety, depression, and post-traumatic stress disorders may occur among front-line medical staff who are in direct contact with the COVID-19 patients (Chersich et al., 2020; Nochaiwong et al., 2020). Moreover, recent studies have demonstrated that the outbreak of COVID-19 had a significant impact on QoL of health care workers (Huang et al., 2020; Suryavanshi et al., 2020).

In facing this international health emergency, researchers strongly advise that everyone pay special attention to health care workers’ mental health and support them during the COVID-19 outbreak (Xiang et al., 2020). Acute stress responses usually occur in the first month after a traumatic event, accompanied by dissociative, re-experiencing, avoidance, and hyperarousal symptoms (Garfin et al., 2015). A study from Toronto demonstrated that health care workers who had been in contact with SARS patients reported a severe acute trauma response (Maunder et al., 2004). Front-line medical staff may report more severe psychological symptoms and worse QoL (An et al., 2020). Pietrzak et al. (2012) found that police who were older and widowed or divorced were more likely to suffer from post-traumatic stress disorder after experiencing traumatic events. In addition, several recent studies have proved that regular physical activity can lead to positive behavioral changes, strengthen the immune system, and reduce negative psychological impacts (Alsalhe et al., 2020; Jiménez-Pavón et al., 2020; Slimani et al., 2020). Although theoretical and empirical evidence suggested that there might be a strong link between acute stress and general health outcomes, acute post-traumatic stress responses have not been well studied in health care workers (Holman et al., 2014; Jeronimus et al., 2019). It is imperative to assess the acute stress responses after a traumatic event to predict long-term health consequences (Dai et al., 2018). Accordingly, it is equally important to investigate the physical and mental health of health care workers during the COVID-19 outbreak. The purpose of our study is as follows: (1) to determine the status of acute stress and QoL in health care workers, (2) to explore the relationship between acute stress and QoL, and (3) to evaluate the influencing factors of acute stress and QoL.

## Materials and Methods

### Sample

Calculations were performed using G-Power statistical software (G^∗^Power Version 3.1.9.7), and the recommended sample size was 280. The inclusion criteria of the study were as follows: (a) people who obtained a certificate of professional qualification, (b) staff on duty in hospitals during the COVID-19 pandemic, (c) and people who volunteer to participate in the research and sign the informed consent form. In total, 525 participants from 15 hospitals were recruited using a convenient sampling method. The participants were divided into three categories according to their occupation: (1) doctors; (2) nurses; (3) auxiliary staff, including technical executives (pharmacists, therapists, dieticians, and so others). Frontline medical staff were defined as individuals who had direct contact with confirmed or suspected cases through diagnosis, treatment, nursing, nosocomial infection control, case sample collection, and pathogen detection. Otherwise, they were classified as non-frontline medical staff.

### Instruments

#### Demographic Characteristics

All participants were required to complete a demographic questionnaire, including gender, age, marital status, occupation, professional title, education level, disease, physical activity level, and work status. Physical activity was defined as aerobic exercise that lasted for at least 30 min per session and was categorized into never, low (1–2 times per week), moderate (3–5 times per week), and high (6 or more times per week).

Participants were invited to answer questions related to COVID-19. They were required to give an honest response to the following questions: a) What is the current pandemic situation in your area? b) Have you been to Wuhan (in the last month)? c) What is your current infection status regarding COVID-19? d) What do you think are your chances of being infected with COVID-19? e) How long do you think the pandemic will last?

#### Acute Stress Response

Acute stress response was measured by the Stanford Acute Stress Reaction Questionnaire (SASRQ); it is a valid research instrument with good reported internal reliability (0.80–0.95) and test-retest reliability (0.69) (Cardeña et al., 2000). Participants were invited to fill out the Chinese version of SASRQ to report whether they had experienced acute stress related to COVID-19. The SASRQ is a 30-item questionnaire that rates acute reactions to trauma on a 5-point Likert scale. It includes four different subscales and three additional questions about the traumatic event, which refers to COVID-19 in our study. The questionnaire consists of the following: dissociative reactions (10 items), re-experiencing of trauma (6 items), avoidance (6 items), hyperarousal (6 items), and impairment in social functioning (2 items). The symptoms are considered positive if a score above three is obtained on at least one item of each subscale (Roberge et al., 2010). A total score (range 0–150) is calculated through the sum of each item, with higher scores implying more serious acute stress.

#### Quality of Life

The Chinese version of the World Health Organization Quality of Life Questionnaire (WHOQoL-BREF) demonstrated good reliability (0.76–0.90) and validity (0.72–0.82); it was used to assess the QoL of hospital employees in this study. This 26-item instrument, rated on a 5-point Likert scale (range 1–5), consists of two questions on general health and four domains: physical health (7 items), psychological well-being (6 items), social relationships (3 items), and environment (8 items). The total score ranges from 26 to 130, with higher scores reflecting a better QoL.

### Procedure

A non-probabilistic and convenience sampling method was conducted. Potential respondents were recruited exclusively through online methods (QQ, Wechat, E-mail, etc.) and were sent the questionnaire link. To reduce the risk of infection during the COVID-19 pandemic, all participants were invited to complete an online self-report questionnaire anonymously by clicking the survey link or scanning the Quick Response code.

### Experimental Design

A cross-sectional descriptive correlational design was conducted on health care workers to assess their acute stress response and QoL during COVID-19. Before recruitment commenced, the study was designed following the Helsinki principles and approved by the Local Ethics Committee of Qianfoshan Hospital Affiliated with Shandong University (2020S517). All respondents provided informed consent (completed online) to participate in the research (10 February to 17 February, 2020). This study is reported as per the STROBE checklist.

### Statistical Analyses

Descriptive statistics were generated for all variables. The continuous demographic data included mean and standard deviation (SD), whereas frequencies and percentages were used to summarize the categorical variables. For each variable, Kolmogorov-Smirnov’s test was utilized to inspect the normality, and Levene’s test was performed to determine the homogeneity of variance. The independent-samples *t*-test (or Mann–Whitney *U*-tests) and the one-way analysis of variance (or Welch’s test) were used to evaluate the differences in continuous variables. The *post hoc* test was performed with Bonferroni correction or Dunnet T3 test, depending on the homogeneity of variance test. Criteria for entry into the multiple linear regression included variables with *p* ≤ 0.10 in univariate analysis (Kang et al., 2015). Subsequently, the bivariate Pearson’s correlation analysis was utilized to determine the correlation between acute stress and QoL. Stepwise multiple regression analysis was used to identify which variables influenced acute stress response and QoL. All statistical analyses were two-sided, and a *p*-value less than 0.05 was defined as statistically significant. All original data were input and calculated by the IBM SPSS ver. 23.0 for Windows (IBM Corporation, Chicago, IL, United States).

## Results

### Sample Characteristics and Distribution of SASRQ and QoL

Among 525 volunteers, 502 completed the questionnaire, of which 47 were excluded because of missing or implausible data. Finally, 455 individuals were included in this study, with a response rate of 95.6% and an effective rate of 86.6%. Sample characteristics of participants, SASRQ, and QoL scores are summarized in Table 1. More than half of the respondents were under 35 years old (64.0%) and had received undergraduate education or above (94.7%). Of the total, 251 (55.2%) thought that the outbreak was under control, 292 (64.2%) believed the pandemic would last more than two months, and 408 (89.7%) thought they were at risk of contracting COVID-19. Regarding the participants’ scores for SASRQ, among the 455 volunteers (356 women) who enrolled in the study, nearly half (48.8%) experienced dissociative reactions; 26.6% reported symptoms of trauma re-experience; 22.6% exhibited avoidance symptoms; 42.4% experienced hyperarousal, and 31.9% suffered from maladaptive behaviors. The mean scores on SASRQ and QoL were 25.88 (SD = 21.84) and 65.60 (SD = 12.60), respectively.

**TABLE 1:** Univariate analysis of acute stress and quality of life with demographic (*n* = 455).

Variables	*n* (%)	Acute stress response			Quality of life		
		Mean ± SD	*t*/*F*	*p* (*post hoc*)	Mean ± SD	*t*/*F*	*p* (*post hoc*)
Gender	−0.913	0.362		0.588	0.557		
Male	99 (21.8)	24.11 ± 23.34			66.26 ± 12.66		
Female	356 (78.2)	26.38 ± 21.41			65.42 ± 12.59		
Age (years)			1.197	0.303		2.406	0.091
≤ 35	291 (64.0)	25.58 ± 21.09			64.65 ± 12.56		
35–60	154 (33.8)	27.07 ± 23.67			67.19 ± 12.50		
>60	10 (2.2)	16.40 ± 8.82			68.85 ± 13.46		
Marital status			4.062	0.018		0.393	0.675
Divorced/Widowed^a^	7 (1.5)	27.86 ± 10.53		a > b, *p* = 0.016^†^	61.53 ± 7.21		
Married^b^	267 (58.7)	22.40 ± 1.37		a > c, *p* = 0.007^†^	65.56 ± 12.12		
Single^c^	181 (39.8)	20.35 ± 1.51			65.82 ± 13.45		
Occupation			0.456	0.634		1.305	0.272
Nurse	229 (50.3)	25.42 ± 21.80			66.33 ± 12.99		
Doctor	162 (35.6)	25.57 ± 21.66			65.41 ± 12.64		
Auxiliary staff	64 (14.1)	28.30 ± 22.60			63.48 ± 10.87		
Professional title			0.053	0.949		1.683	0.187
Primary	282 (62)	25.62 ± 21.08			64.78 ± 12.63		
Intermediate	112 (24.6)	26.26 ± 23.30			67.27 ± 12.27		
Senior	61 (13.4)	26.39 ± 22.86			66.33 ± 12.88		
Educational level			1.334	0.264		1.326	0.266
Associate degree or below	24 (5.3)	24.96 ± 17.97			68.24 ± 12.23		
Bachelor’s degree	212 (46.6)	27.67 ± 23.06			64.69 ± 13.19		
Master’s degree or above	219 (48.1)	24.26 ± 20.94			66.19 ± 12.02		
Chronic disease history			−1.624	0.105		0.416	0.677
Yes	14 (3.1)	16.57 ± 22.73			66.98 ± 11.82		
No	441 (96.9)	26.18 ± 21.77			65.56 ± 12.63		
Physical activity			5.457	0.002			
Never^a^	313 (68.8)	28.28 ± 22.78		a > c, *p* = 0.029^‡^	63.71 ± 12.41	8.072	< 0.001
1–2 times/week^b^	68 (14.9)	21.16 ± 20.68			69.01 ± 11.41		b > a, *p* = 0.001^†^
3–5 times/week^c^	60 (13.2)	21.07 ± 16.67			70.58 ± 11.79		c > a, *p* < 0.001^†^
6 times or more/week^d^	14 (3.1)	15.79 ± 16.11			70.05 ± 16.19		
Front-line medical staff			5.307	<0.001		−6.009	<0.001
Yes	164 (36)	33.61 ± 25.91			61.05 ± 11.56		
No	291 (64)	21.53 ± 17.79			68.17 ± 12.45		
Perceived pandemic status			4.306	0.014		1.027	0.381
Under control^a^	251 (55.2)	22.94 ± 19.19		c > a, *p* = 0.028^‡^	66.36 ± 12.32		
Prevail peak^b^	35 (7.7)	31.43 ± 25.25			66.16 ± 11.06		
Upward trend^c^	90 (19.8)	31.41 ± 25.52			63.75 ± 14.11		
Indetermination^d^	79 (17.4)	26.49 ± 22.30			65.05 ± 12.27		
Have been to Wuhan (in the last month)			2.941	0.003		−1.459	0.145
Yes	14 (3.1)	42.64 ± 25.33			60.77 ± 11.31		
No	441 (96.9)	25.35 ± 21.54			65.76 ± 12.62		
Infection status of COVID-19			1.606	0.206		0.355	0.723
Infected	0 (0)	0			0		
Quarantine	6 (1.3)	14.67 ± 5.85			67.42 ± 7.01		
Uninfected	449 (98.7)	26.03 ± 21.94			65.58 ± 12.66		
Perceived risk of contracting COVID-19			12.698	<0.001		10.477	<0.001
Norisk^a^	47 (10.3)	15.75 ± 18.41		c > a, *p* < 0.001^‡^	71.11 ± 12.55		a > c, *p* < 0.001^†^
Low risk^b^	272 (59.8)	23.06 ± 18.71		c > b, *p* < 0.001^‡^	66.81 ± 12.76		a > d, *p* < 0.001^†^
Medium risk^c^	124 (27.3)	34.15 ± 25.67		d > a, *p* = 0.005^‡^	61.78 ± 1 0.98		b > c, *p* < 0.001^†^
High risk^d^	12 (2.6)	44.25 ± 22.23		d > b, *p* < 0.042^‡^	56.17 ± 10.40		b > d, *p* = 0.003^†^
Expected duration of the pandemic			5.173	0.072		1.014	0.386
1–2 months^a^	163 (35.8)	23.32 ± 19.09			66.55 ± 12.27		
2–3 months^b^	253 (55.6)	26.01 ± 21.35			65.07 ± 12.41		
3–6 months^c^	33 (7.3)	32.49 ± 30.76			66.18 ± 14.91		
≥6 months^d^	6 (1.3)	53.83 ± 32.15			59.08 ± 15.66		

*SD, standard deviation; COVID-19, coronavirus disease 2019. ^†^*p*-value of Bonferroni correction. ^‡^*p*-value of Dunnet T3 test. The variables such as physical activity, perceived pandemic status, perceived risk of contracting COVID-19 and expected duration of the pandemic were divided into four categories: a, b, c, and d, respectively. Marital status was divided into three categories: a, b, and c.*

In the univariate analysis, the acute stress response levels varied significantly among differences in marital status (*F* = 4.062, *p* = 0.018) and physical activity (*F* = 5.457, *p* = 0.002). Acute stress was significantly higher in people who were divorced/widowed and those who were not physically active. The statistical differences in the degrees of acute stress were intimately tied to the perceived risk of contracting COVID-19 (*F* = 12.698, *p* < 0.001) and perceived pandemic status (*F* = 4.306, *p* = 0.014). Participants who perceived a medium or high risk of contracting COVID-19 and perceived an upward trend in the pandemic’s infection rate showed higher scores in SASRQ. Similarly, the front-line medical staff (*t* = 5.307, *p* < 0.001) and people who had been to Wuhan in the last month (*t* = 2.941, *p* = 0.003) were significantly more likely to exhibit acute stress.

Regarding QoL, there was a significant difference in physical activity (*F* = 8.072, *p* < 0.001), work status (*t* = −6.009, *p* < 0.001), and the perceived risk of contracting COVID-19 (*F* = 10.477, *p* < 0.001). The front-line medical staff was more likely to report a worse QoL. Participants who were regularly physically active and those who perceived themselves to be at no or low risk of contracting COVID-19 showed higher QoL scores (Table 1).

### Correlations Among SASRQ and QoL

As shown in Table 2, the study participants’ acute stress response negatively correlated with QoL (*r* = −0.611, *p* < 0.001). Furthermore, the five dimensions of SASRQ significantly and negatively correlated with all QoL dimensions, which exhibited a strong negative association (*r* < −0.60) between acute stress and QoL in health care workers (all *p* < 0.001).

**TABLE 2:** Correlation between acute stress response and quality of life.

Variables	Total score of QoL scale	Physical health	Psychological health	Social relationships	Environment
Total score of SASRQ	−0.611**	−0.586**	−0.546**	−0.417**	−0.549**
Dissociation	−0.571**	−0.540**	−0.522**	−0.394**	−0.503**
Re-experiencing of trauma	−0.529**	−0.519**	−0.450**	−0.354**	−0.493**
Avoidance	−0.492**	−0.475**	−0.452**	−0.315**	−0.447**
Hyperarousal	−0.624**	−0.599**	−0.554**	−0.441**	−0.545**
Impairment in functioning	−0.414**	−0.391**	−0.354**	−0.287**	−0.390**

QoL scale, quality of life scale; SASRQ, Stanford Acute stress Reaction Questionnaire. **p < 0.001 (2-tailed), based on Pearson’s correlation test.

### Factors Influencing Acute Stress and Quality of Life

Stepwise multiple linear regression analysis was conducted to determine the factors that influenced acute stress and overall QoL. Seven variables, which were significant in univariate analysis, were gradually included in the regression model based on the seven hierarchical steps. Finally, all explanatory variables were incorporated into our regression model and summarized in Table 3. With respects to multivariate linear regression analysis, Table 3 revealed the following: marital status (single: β = −0.424, *p* = 0.017; married: β = −0.443, *p* = 0.012); physical activity (3–5 times/week: β = −0.094, *p* = 0.035); front-line medical staff (β = −0.182, *p* < 0.001); perceived risk of contracting COVID-19 (high risk: β = 0.130, *p* = 0.010; medium risk: β = 0.276, *p* < 0.001); and the expected duration of the pandemic (≥6 months: β = 0.095, *p* = 0.035) collectively accounted for 15.5% of the variance of SASRQ (*R*^2^ = 0.184, adjusted *R*^2^ = 0.155). Since the variables in the regression analysis explain only a small part of the variance, it also indicates that there may be other important predictive variables that have not been included, such as pre-existing mental and physical conditions or pre-existing levels of acute stress and QoL. Therefore, further research is needed.

**TABLE 3:** Multiple linear regression analysis of the influencing factors of acute stress response.

Variables	Unstandardized coefficients (B)	Std. error (SE)	Standardized coefficients (β)	*t*	*p*
**Marital status**					
Divorced/Widowed	Reference				
Married	–19.608	7.791	–0.443	–2.517	0.012*
Single	–18.905	7.898	–0.424	–2.394	0.017*
**Physical activity**					
Never	Reference				
1–2 times/week	–5.024	2.791	–0.080	–1.800	0.073
3–5 times/week	–5.911	2.795	–0.094	–2.115	0.035*
6 or more times/week	–9.367	5.528	–0.074	–1.695	0.091
**Front-line medical staff**					
No	Reference				
Yes	–8.275	2.144	–0.182	–3.859	< 0.001**
**Have been to Wuhan (in the last month)**					
No	Reference				
Yes	–10.774	5.982	–0.085	–1.801	0.072
**Perceived pandemic status**					
Under control	Reference				
Prevail peak	3.038	4.022	0.037	0.755	0.451
Upward trend	3.430	2.623	0.063	1.308	0.192
Indetermination	0.546	2.670	0.009	0.205	0.838
**Perceived risk of contracting COVID-19**					
No risk	Reference				
Low risk	6.359	3.244	0.143	1.960	0.051
Medium risk	13.530	3.561	0.276	3.799	< 0.001**
High risk	17.693	6.804	0.130	2.600	0.010*
**Expected duration of the pandemic**					
1–2 months	Reference				
2–3 months	0.004	2.104	0.000	0.002	0.998
3–6 months	6.119	3.992	0.073	1.533	0.126
≥6 months	18.096	8.547	0.095	2.117	0.035*
*R*^2^	0.184				
Adjusted *R*^2^	0.155				

COVID-19, coronavirus disease 2019. *p < 0.05; **p < 0.001.

The dependent variable was computed as QoL. Acute stress response and four significant variables derived from univariate analysis were tested as independent variables. There were four explanatory variables in the final regression model after five hierarchical steps. Table 4 shows the results of the final multiple linear regression model. In our study, falling between 35 and 60 years of age (β = 0.143, *p* < 0.001), physically active 3–5 times per week (β = −0.109, *p* = 0.004), being a front-line medical staff member (β = 0.137, *p* < 0.001), and the total score of SASRQ (β = −0.545, *p* < 0.001) collectively accounted for 41.2% of the variance of QoL (*R*^2^ = 0.425, adjusted *R*^2^ = 0.412). Additionally, acute stress response accounted for most of the variance (Δ*R*^2^ = 0.373, adjusted Δ*R*^2^ = 0.372) (Table 4).

**TABLE 4:** Multiple linear regression analysis of the influencing factors of quality of life.

Variables	Unstandardized coefficients (B)	Std. error (SE)	Standardized coefficients (β)	*t*	*p*
**Age (years)**					
≤35	Reference				
36–60	3.814	1.001	0.143	3.812	< 0.001**
>60	–0.693	3.179	–0.008	–0.218	0.828
**Physical activity**					
Never	Reference				
1–2 times/week	2.436	1.342	0.067	1.816	0.070
3–5 times/week	3.935	1.357	0.109	2.900	0.004*
6 or more times/week	1.449	2.691	0.020	0.539	0.590
**Front-line medical staff**					
No	Reference				
Yes	3.601	1.036	0.137	3.476	0.001*
**Perceived risk of contracting COVID-19**					
No risk	Reference				
Low risk	–1.553	1.545	–0.061	–1.006	0.315
Medium risk	–2.589	1.722	–0.092	–1.504	0.133
High risk	–3.071	3.250	–0.039	–0.945	0.345
Acute stress response (SASRQ)	–0.315	0.022	–0.545	–14.007	< 0.001**
*R*^2^	0.425				
Adjusted *R*^2^	0.412				

COVID-19, coronavirus disease 2019; SASRQ, Stanford Acute stress Reaction Questionnaire. Explained variance of acute stress response: Δ*R*^2^ = 0.373, Adjusted Δ*R*^2^ = 0.372. *p < 0.05; **p < 0.001.

## Discussion

This study aimed to determine the relationship between acute stress and QoL and explore the influencing factors on health care workers during the outbreak of COVID-19. Our study presented that marital status, physical activity, work status, perceived risk of contracting COVID-19, and the expected duration of the pandemic were significantly associated with the acute stress of health care workers. Furthermore, age, physical activity, work status, and acute stress responses significantly affected the QoL of health care workers.

In the multiple linear regression analysis, results indicated that widowed individuals or those who experienced divorce reported more serious acute stress responses. As a traumatic event, divorce or loss of spouse is commonly accompanied by numerous negative consequences and psychological distress. Pérez et al. (2017) observed that people who had experienced negative life events were more likely to be affected by a major traumatic event, showing higher levels of anxiety, depression and post-traumatic stress. Consistent with previous studies (Rosenbaum et al., 2015; Oppizzi and Umberger, 2018), our findings suggested that engagement with moderate physical activity could alleviate the acute stress response. As an auxiliary means to usual care, physical activity has been proven to improve the health conditions caused by PTSD (Rosenbaum et al., 2015; Oppizzi and Umberger, 2018). In a study conducted in New York, Shechter et al. (2020) found that more than half of medical staff reported acute stress since the outbreak of COVID-19, and the most common coping style was physical activity. Based on the above findings, moderate and regular physical activity can help to deal with the psychological problems associated with COVID-19 quarantine.

Our findings suggested that the front-line medical staff exhibited greater levels of acute stress. Wang et al. (2020) highlighted that acute stress disorder is a prominent psychological problem for front-line health professionals. Working on the front-line is an independent risk factor for negative emotions (Lai et al., 2020). Zhou et al. (2020) showed that workload was associated with psychological disturbances in frontline medical staff. However, health care workers with a larger workload are less likely to participate in the survey and are more likely to receive psychological intervention, which may lead to the underestimation of acute stress (Cole et al., 2009; Zhou et al., 2020). Furthermore, the degree of perceived risk regarding contracting COVID-19 was associated with the level of acute stress response. Lin et al. (2007) reported that a medical staff’s self-perceived risk of infection caused by SARS could lead to severe PTSD. A study from Australia showed that the perceived risk of contracting COVID-19 was associated with acute mental health responses (Newby et al., 2020). The high perceived risk not only causes significant psychological distress and intense fear in individuals, but also prompts them to adopt protective measures (Lee et al., 2020; McCloskey and Heymann, 2020). We also demonstrated that a long expectation of disease duration might increase acute stress. Previous studies showed that prolonged exposure to traumatic events usually indicated detrimental effects (Garfin et al., 2015). When faced with emergencies, exposure to continuous, unpredictable threats, and overestimation of negative effects can lead to intense anticipatory anxiety (Grupe and Nitschke, 2013). Meanwhile, the excessive psychological expectation of potential negative stimuli is an important source of stress responses such as anxiety and hopelessness (Simmons et al., 2011). Our findings indicate that effective interventions are necessary to promote health care workers’ mental health. Moderate physical activity and targeted psychological interventions may be practicable.

In our model, factors affecting the QoL of individuals included age (36–60), being a front-line medical staff, physical activity (3–5 times per week), and the extent of acute stress response. Older participants (ages between 35 and 60) had a higher QoL than younger participants (age ≤ 35). Our conclusion is consistent with an air crash observation, which found that older individuals reported a smaller increase in negative effects caused by the MH17 crash than younger participants (Jeronimus et al., 2019). One possible explanation might be that older medical staff have more experience, professional skills, sophisticated coping strategies to deal with risks and crises, and pay less attention to negative information (Piotrkowska et al., 2019). In the current study, people engaged in moderate physical activity reported higher QoL levels than those who never exercised. Our findings are partly consistent with Slimani et al. (2020), who reported that moderate physical activity was positively correlated with all domains of QoL. Similarly, the WHO recommends at least 150 min of moderate exercise per week to improve QoL during the outbreak of COVID-19.

This study also highlighted that the QoL of front-line medical staff was worse than those who were not in direct contact with patients. All health and safety personnel are shown to be at high risk; notably, Lai et al. (2020) showed that the more severe symptoms of depression, anxiety, and insomnia were reported by front-line workers. Moreover, heavy protective equipment and N95 masks make it difficult to breathe and communicate. Prolonged exposure to the virus and the possible risk of infection could increase work-related and psychological stress. Furthermore, front-line medical staff is more likely to encounter patients dying from COVID-19. Research showed that the disposal of corpses results in negative psychological reactions and a poor QoL, which was the case in a sample of earthquake rescuers (Hsiao et al., 2019).

Furthermore, the multiple linear regression analysis showed that the most prominent potential risk factor was acute stress responses, which contributed 37.2% of the variance, while the remaining two factors only represented 4.0% of the variation on QoL. Our findings, along with previous conclusions, indicated that acute stress response was associated with QoL. A study on front-line health professionals during the outbreak of COVID-19 showed that acute stress response led to serious emotional distress and chest pain (Wang et al., 2020). Chaudhury et al. (2015) demonstrated that a history of acute stress increased individuals’ susceptibility to depression by changing molecular activity in the brain. Lefebvre et al. (2020) illustrated an inverse correlation between acute stress and QoL in samples of victims of violent crime and added the evidence that health-related QoL to remain stable within 12 months. Another study emphasized that a serious onset of acute stress was significantly related to depressive disorders and anxiety symptoms; often manifesting a year later for the first time (Bryant et al., 2012). Recurrent, acute stressors can increase the risk of hypertension by activating the stress-mediating autonomic nervous system (Gerin et al., 2012). Continuous fear stimuli are likely to cause abnormal neurocircuitry patterns, resulting in various physiological damages (Olff et al., 2019). In other words, acute stress not only affects the short-term QoL but also threatens long-term health-related outcomes. It is, therefore, imperative to reinforce the awareness of and intervention on the acute stress of health care workers during the duration of the COVID-19 pandemic.

Generally speaking, our research may provide some ideas toward formulating protective measures for health care workers engaged in the COVID-19 pandemic. We recommend that hospital managers pay close attention to the mental health of health care workers, especially front-line medical staff. Professional psychological counseling services and an adequate supply of personal protective equipment are needed to ensure the safety of these health care providers (Banerjee, 2020).

### Limitations

First, all respondents were asked to consider experiences with COVID-19 as a specific stressful event and review the extent to which the epidemic has interfered with their mental health and daily lives – thereby minimizing the effects of pre-existing stress and QoL on the results. Furthermore, due to the sudden outbreak of the COVID-19 pandemic in China, we only conducted a cross-sectional survey and could not assess the psychological status at a baseline. Further longitudinal studies, with an extended follow up, will be needed to determine the causality between the acute stress response and QoL. Second, an online investigation was conducted as everyone was required to be quarantined. Hence, our sample was not based on random selection from all hospital staff. The use of convenience sampling meant that health care workers who were under extreme stress or an extremely high workload would be less likely to participate in the survey, causing selection bias and an underestimation of acute stress and QoL. A more representative sample will be needed to generalize our research results. Lastly, our study is limited to a self-reported questionnaire, which does not include objective data or clinical diagnoses.

## Conclusion

This study displayed health care workers’ acute stress responses and QoL during the outbreak of the COVID-19 pandemic. Factors such as marital status, physical activity, work status, perceived risk of contracting COVID-19, and the expected duration of the pandemic were significantly associated with increased acute stress responses. In addition, younger individuals, lack of physical activity, front-line medical staff, and higher acute stress scores indicated a worse QoL. It is imperative that the physical and mental health of health care workers are improved, to help combat the COVID-19 pandemic. Our findings can help health practitioners and authorities to identify high-risk individuals and provide them with appropriate intervention and timely protection.

## Data Availability Statement

The data analyzed in this study is subject to the following licenses/restrictions: The dataset presented in this article involves 15 hospitals and the participants of this study did not consent to their data being shared. Requests to access these datasets should be directed to CX, abc181818123@163.com.

## Ethics Statement

The studies involving human participants were reviewed and approved by the Local Ethics Committee of Qianfoshan Hospital Affiliated with Shandong University (2020S517). Written informed consent for participation was not required for this study in accordance with the national legislation and the institutional requirements.

## Author Contributions

LZ, RJ, YJ, ML, and RW: study design, data collection, and analysis plan. LZ, RJ, and CX: manuscript writing and revisions for important intellectual content. All authors: statistical analysis and final versions of the manuscript.

## Conflict of Interest

The authors declare that the research was conducted in the absence of any commercial or financial relationships that could be construed as a potential conflict of interest.
